This article has been retracted.

# Oral Administration of GW788388, an Inhibitor of Transforming Growth Factor Beta Signaling, Prevents Heart Fibrosis in Chagas Disease

**DOI:** 10.1371/journal.pntd.0001696

**Published:** 2012-06-12

**Authors:** Fabiane L. de Oliveira, Tania C. Araújo-Jorge, Elen M. de Souza, Gabriel M. de Oliveira, Wim M. Degrave, Jean-Jacques Feige, Sabine Bailly, Mariana C. Waghabi

**Affiliations:** 1 Laboratório de Genômica Funcional e Bioinformática, Instituto Oswaldo Cruz, Fundação Oswaldo Cruz, Rio de Janeiro, Brazil; 2 Laboratório de Biologia Celular, Instituto Oswaldo Cruz, Fundação Oswaldo Cruz, Rio de Janeiro, Brazil; 3 Laboratório de Inovações em Terapias, Ensino e Bioprodutos, Instituto Oswaldo Cruz, Fundação Oswaldo Cruz, Rio de Janeiro, Brazil; 4 INSERM, Unité 1036, Biology of Cancer and Infection, Grenoble, France; 5 UJF-Grenoble 1, Biology of Cancer and Infection, Grenoble, France; 6 CEA, DSV/iRTSV, Biology of Cancer and Infection, Grenoble, France; Federal University of São Paulo, Brazil

## Abstract

**Background:**

Chagas disease induced by *Trypanosoma cruzi* (*T. cruzi*) infection is a major cause of mortality and morbidity affecting the cardiovascular system for which presently available therapies are largely inadequate. Transforming Growth Factor beta (TGFß) has been involved in several regulatory steps of *T. cruzi* invasion and in host tissue fibrosis. GW788388 is a new TGFß type I and type II receptor kinase inhibitor that can be orally administered. In the present work, we studied its effects *in vivo* during the acute phase of experimental Chagas disease.

**Methodology/Principal Findings:**

Male Swiss mice were infected intraperitoneally with 10^4^ trypomastigotes of *T. cruzi* (Y strain) and evaluated clinically. We found that this compound given once 3 days post infection (dpi) significantly decreased parasitemia, increased survival, improved cardiac electrical conduction as measured by PR interval in electrocardiography, and restored connexin43 expression. We could further show that cardiac fibrosis development, evaluated by collagen type I and fibronectin expression, could be inhibited by this compound. Interestingly, we further demonstrated that administration of GW788388 at the end of the acute phase (20 dpi) still significantly increased survival and decreased cardiac fibrosis (evaluated by Masson's trichrome staining and collagen type I expression), in a stage when parasite growth is no more central to this event.

**Conclusion/Significance:**

This work confirms that inhibition of TGFß signaling pathway can be considered as a potential alternative strategy for the treatment of the symptomatic cardiomyopathy found in the acute and chronic phases of Chagas disease.

## Author Summary

Cardiac damage and dysfunction are prominent features in patients with chronic Chagas disease, which is caused by infection with the protozoan parasite *Trypanosoma cruzi* (*T. cruzi*) and affects 10–12 million individuals in South and Central America. Our group previously reported that transforming growth factor beta (TGFß) is implicated in several regulatory aspects of *T. cruzi* invasion and growth and in host tissue fibrosis. In the present work, we evaluated the therapeutic action of an oral inhibitor of TGFß signaling (GW788388) administered during the acute phase of experimental Chagas disease. GW788388 treatment significantly reduced mortality and decreased parasitemia. Electrocardiography showed that GW788388 treatment was effective in protecting the cardiac conduction system, preserving gap junction plaque distribution and avoiding the development of cardiac fibrosis. Inhibition of TGFß signaling in vivo appears to potently decrease *T. cruzi* infection and to prevent heart damage in a preclinical mouse model. This suggests that this class of molecules may represent a new therapeutic tool for acute and chronic Chagas disease that warrants further pre-clinical exploration. Administration of TGFß inhibitors during chronic infection in mouse models should be further evaluated, and future clinical trials should be envisaged.

## Introduction

Chagas disease, caused by the intracellular kinetoplastid parasite *Trypanosoma cruzi*, is a widely spread distributed debilitating human illness, affecting 10–12 million people in Central and South America. It is a major cause of mortality and morbidity, killing 15,000 persons each year [1], [2]. Chagas disease presents an acute phase of infection that is characterized by mild clinical symptoms (fever and malaise) and high parasitemia, but is often unmarked. Due to a potent specific immune response which control parasitemia, patients usually attain the indeterminate stage of the infection, with low-level of parasite persistence that can last from 10 to 40 years. About one in three infected individuals develops the symptomatic chronic stage of infection, which is characterized mainly by myocardiopathy or/and intestinal megasyndrome. A century has passed since the discovery of Chagas disease and the development of an efficient drug is still a challenge. As other neglected diseases, it has not received much attention of the pharmaceutical industry and present available therapies are insufficient [3]. Nifurtimox and benznidazole, the only two trypanocide drugs available, have toxic side effects, are not effective for all parasite strains and the effect in human chronic phase is still under clinical trial [4]. Moreover, no therapeutic approach targeting Chagas disease heart fibrosis is presently available.

Transforming Growth Factor ß1 (TGFß1) is the prototypic member of a family of polypeptide growth and differentiation factors that play a great variety of biological roles in such diverse processes as inflammation, fibrosis, immune suppression, cell proliferation, cell differentiation, and cell death [5], [6]. TGFß is also involved in many direct and indirect interactions between infectious agents and their hosts [7]. Several studies have demonstrated that TGFß plays a major role in the establishment and pathogenesis of *T. cruzi* infection (reviewed in [8]). Moreover, significantly higher circulating levels of TGFß1 have been observed in patients with Chagas disease cardiomyopathy [9] and in a culture system of cardiomyocytes infected by *T. cruzi* [10]. In order to establish its biological functions, TGFß must be activated into a mature form mainly by proteases, allowing its interaction with a specific transmembrane receptor called TGFß receptor-II (TßRII), which phosphorylates and stimulates the serine/threonine kinase activity of TßRI, also called activin receptor-like kinase 5 (ALK5). Upon activation, ALK5 phosphorylates the cytoplasmic signaling proteins Smad-2 and -3, which then associate with Smad-4, translocate into the nucleus as a multiprotein complex, and stimulate the transcription of TGFß-responsive genes, thereby inducing specific biological responses.

We have recently described that the ALK5 inhibitor, 4-(5-benzo[1,3]dioxol-5-yl-4- pyridin-2-yl-1H-imidazol-2-yl)-benzamide (SB431542) reduces the infection of cardiomyocytes by *T. cruzi in vitro* [11] and we could further show that it also inhibited *T. cruzi* infection *in vivo* and prevented heart damage in a mouse model [12]. This work therefore clearly demonstrated that blocking the TGFß signaling pathway could be a new therapeutical approach in the treatment of Chagas disease heart pathology. However the limitation of this compound was the preclusion to oral administration and some toxic effects. To reinforce the prove of concept, the aim of the present work was therefore to test, in the same parasite-mouse model of experimental Chagas disease, another inhibitor of the TGFß signaling pathway, 4-(4-[3-(Pyridin-2-yl)-1H-pyrazol-4-yl] pyridin-2-yl)-N-(tetrahydro-2Hpyran-4-yl) benzamide (GW788388) which can be orally administered and that has an improved pharmacokinetic profile [13], [14]. We found that GW788388 added 3-day post infection (dpi) decreased parasitemia, increased survival, prevented heart damage, and decreased heart fibrosis. Very importantly, we also demonstrated here for the first time that when added after the end of the intense parasite growth and consequent metabolic shock phase at 20 dpi, GW788388 could still decrease mortality and heart fibrosis.

## Methods

### Parasites

Bloodstream trypomastigotes of the Y strain were used and harvested by heart puncture from *T. cruzi-*infected Swiss mice at the parasitemia peak, as described previously [15].

### Ethics statement

Mice were housed for at least one week before parasite infection at the Animal Experimentation Section at the Laboratory of Innovations in Therapies, Education and Bioproducts-IOC/FIOCRUZ under environmental factors and sanitation according to “Guide for the Care and Use of Laboratory Animals”. Animal studies adhered to the International guidelines (National Research Council. 1996, National Academy press, Washington, DC). This project was approved by the FIOCRUZ Committee of Ethics in Research (protocol number 028/09).

#### In vivo infection

Male Swiss mice (age 6–8 weeks, weight 18–20 g) were obtained from the animal facilities of CECAL (FIOCRUZ, Rio de Janeiro, Brazil). Infection was performed by intraperitoneal (IP) injection of 10^4^ bloodstream trypomastigotes. Age-matched non-infected mice were maintained under identical conditions.

#### Experimental groups

The animals were divided into the following groups: non-infected (NI), infected and untreated (Y DMSO), infected and treated with 3 mg/kg GW783388 (Y GW788388). Ten mice from each group were used for analysis at each different dpi and 5 independent experiments were performed.

#### Drug and treatment

The compound GW783388 (GlaxoSmithkline, France) or vehicle dilution buffer (4% DMSO, 96% [0.5% Hydroxypropylmethylcellulose (HPMC), 5% Tween 20, 20% HCl 1 M in NaH2PO4 0.1 M]) was used for oral administration. Mice received GW788388 at 3 mg/kg at 3 dpi or 20 dpi by gavage in a single administration (0.2 mL). The control group received vehicle buffer using the same schedule.

#### Survival rates and parasitemia

Parasitemia was individually checked by direct microscopic counting of parasites in 5 µL of blood, as previously described [15]. Mortality was checked daily until 30 dpi and expressed as percentage of survival.

#### Biochemistry

Blood was collected from the tip of mice tails of all experimental groups at 15 dpi and immediately analyzed for the determination of aspartate aminotransferase (AST), alanine aminotransferase (ALT) and urea levels with Reflotron Plus (Roche), according to the manufacturer recommendations. ALT and AST activities were used to evaluate hepatic dysfunction and the results were expressed as enzyme concentration (mg/dL). ALT and AST belong to the group of transaminase that catalyses the conversion of amino acids into corresponding α-ceto acids and vice-versa by transference of amine groups. Urea was measured to evaluate renal function and the results were expressed in concentration (mg/dL).

#### Histopathology

Fixed tissue was dehydrated and embedded in paraffin. Sections (3 µm) stained by routine haematoxylin-eosin (HE) were analyzed by light microscopy. The number of amastigote nests and of inflammatory infiltrates (more than 10 mononuclear cells), were determined in 30 microscopic fields/slide (total magnification, 400×). The mean number of amastigotes or inflammatory infiltrates per field was obtained at 15 dpi from at least three infected mice, with three sections per mouse per group. The sections were observed using a Zeiss Axioplan microscope (Zeiss, Oberkochen, Germany) coupled with Axiovision image acquisition system (Zeiss). The area (%) of inflammatory infiltrates was evaluated using NIH ImageJ software in at least 10 images per group.

#### Histological assessment of cardiac fibrosis

Heart fibrosis was studied by (a) Masson's trichrome staining at 15, 20 and 24 dpi as previously described [16], (b) immunohistochemical staining of specific extracellular matrix proteins (collagen type I and fibronectin, see below), and (c) Western blot analysis of collagen type I and fibronectin protein levels (see below). For collagen type I and fibronectin immunostainings, fixed tissue slides were obtained as described above and heart fibrosis was studied by collagen type I and fibronectin immunostainings at 15 dpi. Briefly, after blocking with 3% BSA for 1 hour, the following primary antibodies were applied overnight to the sections: rabbit polyclonal anti-collagen type I (Novotec, France, kindly provided by Dr. Daniella Areas Mendes-da-Cruz, IOC/Fiocruz) and rabbit polyclonal anti-fibronectin (Sigma Aldrich, USA). The secondary antibody was Alexa 594 goat anti-rabbit IgG (Invitrogen). Negative control sections were incubated with non-immune rabbit serum and the secondary antibody alone and indicated no cross reactivity (data not shown). Host-cell nuclei were stained with 4′,6-diamidino-2-phenylindole dihydrochloride (DAPI). The sections were observed using a Zeiss Axioplan microscope (Zeiss) coupled with Axiovision image acquisition systems (Zeiss). Subsequent automated analysis of the captured images (6–10 mice per group) was carried out using an ImageJ macrobased algorithm that identifies, separates and quantifies the light blue areas stained with Masson's trichrome representing fibrosis.

#### Cx43 plaque quantification

Cx43 staining on fixed tissue was performed as described above. Briefly, heart sections were blocked with 3% BSA for 1 hour, and incubated overnight with rabbit polyclonal anti-connexin 43 (Sigma Aldrich, USA). The secondary antibody was Alexa 488 goat anti-rabbit IgG (Invitrogen). Host-cell nuclei were stained with DAPI. The images were obtained using a Zeiss Axioplan microscope at final magnification of ×400. At this magnification, a typical test area included approximately 34.600 µm^2^ of tissue area. The images obtained in each studied case were analyzed using the NIH software ImageJ to determine the mean number and the length of Cx43 plaques by quantification of 3-field images/animal.

#### Immunoblot analysis

Left ventricular heart proteins from each group (NI, Y DMSO and Y GW788388) were extracted from 100 mg tissue/mL phosphate-buffered saline, to which 0.4 mol/L sodium chloride, 0.05% Tween 20, and protease inhibitors (0.1 mmol/L phenylmethylsulfonyl fluoride and 1/100 protease inhibitors cocktail (Sigma)) were added. The samples were sonicated twice and centrifuged for 10 min at 3000 *g*, and the supernatant was kept frozen at −70°C. Proteins in the lysates (20 µg/lane) were separated by SDS/PAGE and analyzed by immunoblotting with specific primary antibodies (rabbit Anti-fibronectin and rabbit Anti-connexin-43 from Sigma Aldrich and rabbit Anti-collagen type I from Novotec, France). To confirm equal protein loading, the same membranes were stripped and reprobed with a monoclonal antibody against GAPDH (Pierce).

#### Electrocardiography (ECG)

ECG recording and analysis were performed in the three groups, as reported (30). Briefly, mice were fixed in the supine position, and transducers were carefully placed on the skin in accordance to chosen preferential derivation (lead II). Traces were recorded using a digital system (Power Lab 2/20) connected to a bio-amplifier in 2 mV for 1 s (PanLab Instruments). Filters were standardized between 0.1 and 100 Hz and traces were analyzed using the Scope software for Windows V3.6.10 (PanLab Instruments). ECG parameters were evaluated in the acute phase at 15 dpi, using the following standard criteria: (i) the heart rate, monitored by beats/minute (bpm), and (ii) the variation at P wave and PR, QRS and QT intervals, all measured in milliseconds (ms).

#### Statistical analysis

Differences were considered statistically significant when p<0.05 (*) or p<0.01 (**), as determined by GraphPadPrism 4.0 software (Graph- Pad Software Inc., San Diego, CA, USA). The Kaplan- Meier test was used to analyze the significances of the survival rates while all the other analyses were performed using the non-parametric Mann–Whitney test.

## Results

The aim of the present work was to evaluate whether the compound GW788388, which is an ATP-competitive inhibitor of the kinase activity of ALK5, could have a beneficial effect *in vivo* in an experimental model of mouse acute infection by *T. cruzi* and whether it could protect infected mice from parasite-induced alterations of cardiac functions and fibrosis when administrated early (3 dpi) and late (20 dpi).

### Oral administration of GW788388 at 3 dpi reduced parasitemia and heart damage and increased mice survival rates in *T. cruzi*-infected mice

In the first set of experiments, the inhibitor GW788388 was orally administered to male Swiss mice infected with 10^4^ bloodstream trypomastigotes of the Y strain (day 0), at the 3rd dpi. We first performed a dose-response study by administering different doses of GW788388 (0.3, 3, 6 and 15 mg/kg) and analyzed parasitemia and survival rate. The results showed a dose-dependent inhibition of parasitemia at 8 dpi from 0.3 to 15 mg/kg of GW788388 (Methods S1 and Fig. S1A). On the other hand, the survival rate was increased with 3 or 6 mg/kg of GW788388 but unaltered at 0.3 and 15 mg/kg, suggesting some toxicity of the drug at this largest dose (Fig. S1B). For the subsequent studies, the dose of 3 mg/kg was chosen since it was the lowest GW788388 concentration that significantly affected parasitemia without worsening mortality. The choice for 3 mg/kg GW788388 administration was further reinforced by the assays performed by Gellibert and collaborators [13], who showed in a model of kidney fibrosis that doses as low as 3 mg/kg/mice of GW788388 significantly inhibited collagen type I mRNA levels. The control group received the vehicle buffer in which GW788388 was diluted (4% DMSO, 96% [0.5% Hydroxypropylmethylcellulose (HPMC), 5% Tween 20, 20% HCl 1 M in NaH2PO4 0.1 M]) and could be considered as the placebo group. The responses of DMSO-treated infected mice were not significantly different from those of untreated infected mice, excluding any sham or placebo effect (data not shown). In our model of acute infection, as previously described [12], parasitemia peaked at 8 dpi (Fig. 1A). We found that GW788388 administration at 3 dpi significantly reduced the blood parasitemia peak (Fig. 1A). Further, as previously described with the compound SB421543 [11], we could demonstrate that *in vitro* administration of GW788388 on cardiomyocytes impaired *T. cruzi* replication in host cells (Fig. S2) supporting the decreased parasitemia peak found *in vivo*. On the other hand, no effect of GW788388 on trypomastigote forms of *T. cruzi* viability could be observed after direct incubation of the drug with the parasites (unpublished result). We also showed that GW788388 administration significantly increased survival rates at 30 dpi (65% in the treated-group versus 34% in the untreated group, Fig. 1B). The infection induced a loss of body weight at 14 dpi [12], which was not modified by the administration of GW788388 (data not shown). To investigate whether GW788388 treatment would also affect myocardial parasitism and infiltration of inflammatory cells, we analyzed mouse infected heart sections collected at 15 dpi using histochemical techniques. Non-infected animals showed no inflammatory infiltration in the myocardium (data not shown). Myocardial sections from the *T. cruzi*-infected sham-treated group (Y DMSO) had many amastigote nests (Fig. 1C, open arrows) and large inflammatory foci (Fig. 1E, filled arrows) that were frequently associated with fibrotic areas. GW788388 treatment significantly decreased the number of amastigote nests (Fig. 1D and 1G). GW788388 administration also significantly decreased the area invaded by inflammatory infiltrates (Fig. 1F and 1H). A more detailed count of the number of cells per inflammatory foci showed that GW788388 treatment more particularly decreased the number of large inflammatory foci within the myocardium (larger than 20 or 50 cells per inflammatory infiltrates) (Table 1).

**Figure 1:** GW788388 administration at 3 dpi decreased parasitemia and heart inflammatory infiltrates and increased survival rates. Male Swiss mice were injected IP with 10^4^ bloodstream trypomastigotes. Then GW788388 (3 mg/kg) or DMSO was administered by gavage at 3 dpi. (A) Parasitemia was measured by direct counting of parasites in blood. (B) Percent survival was monitored during the experiment until 30 dpi. (C–F) At 15 dpi, mice were sacrificed and heart sections stained with hematoxylin-eosin were analyzed by light microscopy. Numerous amastigote nests (C, open arrows) and large inflammatory infiltrates (E, filled arrows) were observed in untreated *T. cruzi*-infected mice. GW788388 administration decreased the number of amastigote nests (D, open arrow) and of inflammatory infiltrates (F). (G and H) The mean number of amastigote nests in 30 fields (G) and the area (%) of inflammatory infiltrates (more than 10 mononuclear cells) (H) are shown. Values for the infected group treated with GW788388 that were significantly different from the value for the DMSO infected group are indicated (**p<0.01 and * *p<*0.05). n = 10 mice/group in 4 independent experiments.

**Table 1:** Effect of GW788388 on the number of inflammatory infiltrates in the heart at 15 dpi.

Number of cells per Inflammatory Infiltrates	Y DMSO	Y GW788388	Fold decrease	*P* value
Total	168±45	94±29	1.78	0.008^a^
>50	29±18	4±2	6.07	0.004^a^
21–50	66±19	24±10	2.75	0.002^a^
10–20	73±28	65±18	1.12	0.68

*T. cruzi* infected mice were treated with 3 mg/kg GW788388 at 3 dpi and the number of inflammatory infiltrates in the heart was counted at 15 dpi.

a Significant differences (*p*<0.01) between the values for infected non treated (Y DMSO) and treated (Y GW788388) groups of mice.

### GW788388 controlled liver alteration caused by acute experimental *T. cruzi* infection

*T. cruzi* infection induces a strong hepatitis during the acute phase of Chagas disease [17]. We therefore analyzed several parameters of the liver in sham-treated versus GW788388-treated mice. Analysis of liver sections at 15 dpi revealed the presence of large inflammatory infiltrates in DMSO-treated animals (Fig. 2A, arrow). GW788388 administration significantly decreased the number of these infiltrates (Fig. 2B and C). We also measured two circulating markers of hepatic function which are induced by *T. cruzi* infection: AST (aspartate aminotransferase) and ALT (alanine aminotransferase). We found that GW788388 administration significantly decreased the serum levels of AST and ALT (Fig. 2D and E). We also measured urea, which reflects the renal functional status. Urea level was significantly increased at 15 dpi in DMSO-treated animals while GW788388 administration significantly reduced it (Fig. 2F).

**Figure 2:** GW788388 administration at 3 dpi decreased liver and renal alterations. Male Swiss mice were injected IP with or without (NI) 10^4^ bloodstream trypomastigotes. Then GW788388 (3 mg/kg) or DMSO was administered by gavage at 3 dpi. (A and B) At 15 dpi mice were sacrificed, and liver sections stained with hematoxylin-eosin were analyzed by light microscopy. Large inflammatory infiltrates (A, white arrow) were observed in untreated *T. cruzi*-infected mice. (C) The mean number of inflammatory infiltrates (more than 10 mononuclear cells) in 30 fields is shown. (D and E) The serum levels of AST and ALT, two markers of hepatic lesion, were measured at 15 dpi. (F) The serum urea levels were measured to evaluate renal function. Each symbol shows the value for one mouse. The short black bars show the mean value for each group. Values that were significantly different from studied groups are indicated by asterisks (**p<0.01 and * *p<*0.05). n = 3 mice/group in 3 independent experiments.

### GW788388 prevented heart damage from *T. cruzi* infection

We next analyzed electrocardiograms (ECG) of the different groups of mice at 15 dpi. As expected, analysis of the ECG demonstrated an atrial ventricular block with PR interval higher than 40 ms, leading to sinus bradycardia in sham-treated *T. cruzi*-infected animals as compared to the non-infected control group (495.8 and 774.2 bpm, respectively, Figure 3 and Table 2). GW788388 administration significantly limited the bpm decrease at 15 dpi, with a mean heart rate of 554.3 (Fig. 3 and Table 2). The other parameters analyzed demonstrated that infected mice had higher QT, PR and QRS intervals compared to non-infected mice (Table 2), and that GW788388 administration (3 mg/kg) also significantly decreased the QT intervals to 25.3 ms as compared to 29.6 in the infected DMSO-treated group (Table 2). A possible cause of this worsening in heart electrical conduction after the infection could be the direct effect of TGFß in heart cells. It has been already proposed that elevated TGFß levels during *T. cruzi* infection disorganize gap junctions, possibly contributing to abnormal impulse conduction and arrhythmia in Chagas disease [12]. To test this hypothesis, we measured connexin 43 (Cx43) expression in the different groups of mice. Heart sections from at least three mice per group at 15 dpi were immunostained for Cx43. We observed by confocal microscopy that non-infected hearts presented a dense structure of gap junction plaques (Fig. 4A, green staining). A drastic change in Cx43 expression was observed in the infected hearts of vehicle-treated mice, with an important decrease in Cx43 expression and a disruption of gap junction plaques (Fig. 4B). We found that GW788388 treatment reduced Cx43 disassembly and prevented the dissolution of gap junctions, preserving organized plaque distribution (Fig. 4C). The mean number of Cx43 plaques and their mean length were significantly lower in the heart of infected mice at 15 dpi as compared to the non-infected group (Fig. 4D and E). GW788388 treatment protected infected-mice from this loss as the decrease in the mean number of plaques was only reduced by 30% versus 45% in non-treated mice (Fig. 4D) and the mean length was similar to the non-infected mice (Fig. 4E). Immunoblotting analysis of Cx43 expression from heart ventricles confirmed these data (Fig. 4F and G).

**Figure 3:** GW788388 administration at 3 dpi restored Electrocardiographic parameters. Male Swiss mice were injected IP with or without (NI) 10^4^ bloodstream trypomastigotes. Then GW788388 (3 mg/kg) (Y GW788388) or DMSO (Y DMSO) was administered by gavage at 3 dpi. Representative electrocardiographic tracings of the three groups at 15 dpi are shown. n = 6 mice/group in 3 independent experiments.

**Figure 4:** GW788388 administration at 3 dpi inhibited connexin 43 disruption. Male Swiss mice were injected IP with or without (NI) 10^4^ bloodstream trypomastigotes. Then GW788388 (3 mg/kg) (Y GW788388) or DMSO (Y DMSO) was administered by gavage at 3 dpi. (A–C) At 15 dpi, mice were sacrificed and heart sections stained with anti-Cx43 antibody (green, Cx43 plaques are indicated by white arrows) and DAPI (nuclei, colored in blue). Quantitative analysis of the number of Cx43 plaques (D) and length (E), on images from each group studied (NI, Y DMSO and Y GW788388). Values are expressed as the mean±SD (F) 20 µg of total proteins from hearts at 15 dpi were resolved in 12% SDS/PAGE and immunoblotted with anti-Cx43 and glyceraldehyde-3-phosphate dehydrogenase (GAPDH) antibodies. (G) Densitometric histograms of the normalized levels of Cx43 as related to GAPDH are shown. Values that were significantly different from studied groups are indicated by asterisks (* *p<*0.05). n = 3 mice/group in 3 independent experiments.

**Table 2:** Effect of GW788388 on electrocardiograph parameters at 15 dpi.

ECG parameters (Mean ± SD)	Non-infected	Y + DMSO	Y + GW788388
Heart rate (bpm)	774.2±30.6	495.8±79.2^a^	554.3±44.5^c^
PR intervals (ms)	28.6±3.1	50.4±8.2^a^	45.1±8.4
QRS intervals (ms)	8.6±1.4	10.6±2.7^b^	9.7±2.0
QT intervals (ms)	22.8±8.9	29.6±5.5^b^	25.3±6.4^c^
Frequency of AVB1	0/10 (0%)	15/18 (83%)	5/18 (28%)
Frequency of AVB2	0/10 (0%)	13/18 (72%)	6/18 (33%)

ECG parameters were evaluated in the acute phase at 15 dpi, using the following standard criteria: (i) the heart rate was monitored by beats/minute (bpm), and (ii) the variation at P wave and PR, QRS and QT intervals, all measured in milliseconds (ms). The incidence of AVB1, atrioventricular block type 1 and AVB2, atrioventricular block type 2 are stated in absolute numbers and in percentage. Significant differences between the values for non-infected and infected groups of mice:

a (*p*<0.01) and.

b (*p*<0.05).

c Significant differences (*p*<0.05) between the values for infected non treated (Y DMSO) and treated (Y GW788388) groups of mice.

### GW788388 prevented heart fibrosis development in *T. cruzi*-infected mice

One of the best established biological function of TGFß is the stimulation of extracellular matrix (ECM) protein deposition. Therefore, we checked whether GW788388 treatment would affect heart fibrosis that occurs in response to *T. cruzi* infection. Left ventricular heart tissues were obtained from each group and the deposition of ECM proteins was studied by immunostaining for collagen type I and fibronectin at 15 dpi. We observed an interstitial fibrous heart with high levels of both collagen type I and fibronectin deposition, as observed in red on Figure 5A and C, respectively. Interestingly, we could show that oral administration of GW788388 significantly reduced collagen type I and fibronectin levels (Fig. 5B and D, respectively). These data were confirmed by immunoblotting analysis of collagen type I and fibronectin expression from heart ventricles (Fig. 5E, F and G).

**Figure 5:** GW788388 administration at 3 dpi decreased heart fibrosis. Male Swiss mice were injected IP with or without (NI) 10^4^ bloodstream trypomastigotes. Then GW788388 (3 mg/kg) (Y GW788388) or DMSO (Y DMSO) was administered by gavage at 3 dpi. At 15 dpi, mice were sacrificed and heart sections stained with anti-collagen type I antibody (A and B, open arrow) or anti-fibronectin antibody (C and D, white arrow) colored in red and DAPI (nuclei, colored in blue). (E) 20 µg of total proteins from hearts at 15 dpi were resolved in 12% SDS/PAGE and immunoblotted with anti-fibronectin or anti-collagen type I antibodies and reprobed with anti-glyceraldehyde-3-phosphate dehydrogenase (GAPDH) antibody. (F and G) Densitometric histograms of the normalized levels of fibronectin or collagen type I as related to GAPDH are shown. Values that were significantly different from studied groups are indicated by asterisks (**p<0.01 and * *p<*0.05). n = 3 mice/group in 3 independent experiments.

We found that GW788388-treatment decreased the phosphorylation level of Smad2 in infected hearts, demonstrating that GW788388-treatment was related to TGFß dependent signaling in vivo (data not shown).

### Oral administration of GW788388 at 20 dpi also increased mice survival rates and reduced heart fibrosis in *T. cruzi* infected mice

Because most of the beneficial effects that we observed here with the TGFß inhibitor (GW788388) might be due to the resulting decreased parasitemia due to the inhibitory effect of TGFß signaling inhibitors in host cell invasion and intracellular proliferation [11], [12], we next studied the effect of GW788388 oral administration after the parasitemia peak. We chose to add GW788388 at 20 dpi as by this time, only 18% of infected mice survived and 30% of them died at 24 dpi. Interestingly, we found that GW788388 administration at 20 dpi completely protected these mice (n = 12) from death until 24 dpi (Fig. 6A, inset). In the inset, 100 represents the percentage of survival rate calculated from 20 dpi. GW788388 administration still decreased the number of inflammatory infiltrates within the myocardium (Table 3). To verify if GW788388 treatment presented an effect in the reversion of installed fibrosis, we performed Masson's trichrome staining on heart cross-sections of infected untreated mice at 15 dpi (Fig. 6B), 20 dpi (Fig. 6C) and 24 dpi (Fig. 6D), and of infected GW788388-treated mice at 24 dpi (Fig. 6E). We observed a progressive increase in collagen deposition visualized as light blue staining, which followed fibrosis progression (from 15 to 24 dpi, Table 4). At 20 dpi, which corresponded to the day of GW788388 administration, we observed a fibrotic pattern on the heart of infected mice frequently associated to inflammatory infiltrates (Fig. 6C). Interestingly, four days after GW788388 administration (i.e. 24 dpi) we observed a decrease in collagen deposition (Fig. 6E) as compared to the untreated group (Fig. 6D, Table 4). Immunoblotting assays were performed to compare the expression levels of collagen type I between each group. We observed a significant increase in collagen type I expression in the DMSO infected group as compared to the non-infected group (Fig. 6F and G, 9 fold increase), while GW788388 administration to infected mice significantly decreased the expression levels of collagen type I (Fig. 6F and G).

**Figure 6:** GW788388 administration at 20 dpi protected *T. cruzi*-infected mice from death and decreased heart fibrosis. Male Swiss mice were injected IP with or without (NI) 10^4^ bloodstream trypomastigotes. Then GW788388 (3 mg/kg) (Y GW788388) or DMSO (Y DMSO) was administered by gavage at 20 dpi. (A) Percent survival was monitored during the experiment until 24 dpi (Inset shows a blow-up of the survival curve from 20 to 24 dpi (100 represents the percentage of survival calculated from 20 dpi)). (B, C, D, E) Untreated infected mice were sacrificed at 15 dpi (B), 20 dpi (C), 24 dpi (D) and GW788388-treated mice at 20 dpi were sacrificed at 24 dpi (E). Heart sections were stained for collagen deposition by Masson's trichrome (light blue staining, open arrows). (F) 20 µg of total proteins from hearts at 24 dpi were resolved in 12% SDS/PAGE and immunoblotted with anti-collagen type I antibody and reprobed with anti-glyceraldehyde-3-phosphate dehydrogenase (GAPDH) antibody. (G) Densitometric histograms of the normalized levels of collagen type I as related to GAPDH are shown. Values that were significantly different from studied groups are indicated by asterisks (**p<0.01 and * *p<*0.05). n = 4 mice/group in 3 independent experiments.

**Table 3:** Effect of GW788388 on the number of inflammatory infiltrates in the heart at 24 dpi.

Number of cells per Inflammatory Infiltrates	Y DMSO	Y GW788388	Fold decrease	*P* value
10–20	40±4	27±5	1.5	0.02^a^
21–50	14±6	9±4	1.5	0.3
>50	11±7	2±1	4.3	0.1
Total	66±18	39±5	1.7	0.1

*T. cruzi* infected mice were treated with 3 mg/kg GW788388 at 20 dpi and the number of inflammatory infiltrates in the heart was counted at 24 dpi.

a Significant differences (*p*<0.05) between the values for infected non treated (Y DMSO) and treated (Y GW788388) groups of mice.

**Table 4:** Effect of GW788388 on the fibrosis scores of the heart at 20 dpi.

	dpi 15 DMSO	dpi 20 DMSO	dpi 24 DMSO	dpi 24 GW788388
Number of mice	7	8	10	6
% area stained for Masson' Trichrome	25.7	33.8	55.8	4.8
	23.9	18.8	35.7	6.2
	22.6	14.4	30.0	3.1
	5.2	53.8	7.7	2.9
	56.1	55.9	8.2	2.9
	5.1	13.2	13.7	8.3
	nd	39.4	54.0	
		16.1	54.0	
			20.2	
			9.2	
Mean ± SD	23.1±18.6	30.7±17.6	28.9±20.0	4.7±2.2**

*T. cruzi* infected mice were treated with 3 mg/kg GW788388 at 20 dpi and fibrosis was quantified before (15 and 20 dpi) and after (24 dpi) treatment. Percent of Masson's Trichrome stained area (light blue areas) were quantified using NIH ImageJ Software in the microscopic images of heart sections.

**: Significant differences (*p*<0.01) between the values for Y DMSO and Y GW788388 groups of mice observed at 24 dpi. nd: not detected.

## Discussion

We have recently demonstrated that *in vivo* inhibition of the TGFß signaling pathway can decrease infection and prevent heart damage [12], suggesting that this new class of therapeutic agents should be considered in association with trypanocidal compounds for the potential treatment of Chagas disease cardiomyopathy. In the present work, we demonstrated that a more potent inhibitor of the TGFß signaling pathway, GW788388, which can be orally administered, significantly decreased parasitemia, increased survival and restored cardiac function as measured by ECG heart frequency (increase in bmp) and atrial conduction (decrease in QT interval). When administered at 3 dpi, we observed that GW788388 treatment reduced parasitemia and its subsequent deleterious effects. Whether the protective effect of GW788388 results only from this sole anti-infectious effect remains to be established. However, the short half-life of GW788388 in vivo (plasma T1/2 = 1.3 hours; [13]) makes it unlikely that it is mediated by long-term effects on e.g. fibrosis or cardiac rhythm. In contrast, administration of GW788388 at 20 dpi to mice that survived the metabolic distress syndrome clearly resulted in improved survival, which correlated with decreased cardiac fibrosis and has probably no causal relationship with the anti-infectious effect of the drug. Given the recent availability of reliable mouse models for chronic chagasic cardiomyopathy [18], the present proof that orally administrated GW788388 is feasible and efficient in the acute phase will offer in the near future the possibility of testing TGFß inhibitors in the chronic phase in pre-clinical assays. Taken together, these data further support that blocking TGFß signaling could represent a potential new therapeutic approach for Chagas disease heart fibrosis treatment.

It is now well established that the involvement of the TGFß signaling pathway plays an important role in the development of Chagas disease [8]. TGFß has been shown to be involved during parasite-host cell invasion, proliferation and differentiation [19]–[22]. Moreover, significantly higher circulating levels of TGFß1 have been observed in patients with Chagas disease cardiomyopathy [9], [16]. These data incited us to test the possibility of treating the development of Chagas disease by blocking the TGFß signaling pathway.

Here, we show that oral administration of GW788388 kinase signaling inhibitor prevents parasitemia, mortality, and heart fibrosis to acutely *T. cruzi*-infected mice in comparison to untreated-infected experimental group of animals. In lack of demonstration of GW788388 direct killing effect upon *T. cruzi*, we postulate the protein kinase inhibitor used may induce intracellular parasite latency [23], [24], such as that involved with the Plasmodium sporozoites cell cycle inhibition of initiation factor-2alpha (elF2alpha) kinase (IK2); its down-regulation by removal of PO4 from elF2alpha-P gives rise to the latency [25], [26]. In this regard, ongoing investigations in chronically *T. cruzi*-infected mouse model will determine whether GW788388 beneficial effects can be explained by the drug-induced parasite latency and long lasting cryptic infections.

Several approaches have been developed to abrogate TGFß signaling. Antibodies directed against TGFß have been administered in diabetic rodents and this was shown to efficiently prevent glomerulosclerosis and renal insufficiency [27]. Antisense TGFß oligonucleotides were found to reduce kidney weight in diabetic mice [28]. Recently, a soluble fusion protein of TßRII was reported to reduce albuminuria in a chemically induced model of diabetic nephropathy in rats [29]. And finally, inhibitors of the kinase activity of the TßRI (ALK5) have been developed. These inhibitors interact with the ALK5 ATP-binding site, thereby preventing TGFß intracellular pathways [30]. The first ALK5 inhibitor described, SB431542, is an ATP-competitive kinase inhibitor [31]. SB431542 significantly reduced procollagen1alpha (I) in rat kidneys in a model of induced nephritis. It was also described that SB431542 triggers antitumor activity in vivo [32]. Our work also demonstrated that SB431542 reduced mortality, decreased parasitemia and prevented heart damage as observed by histological and ECG analysis during the acute phase of experimental Chagas disease [12]. However, the limitations of SB431542 were the need of intraperitoneal injection and the *in vivo* toxic effects that have been demonstrated. Recently, GW788388 was developed as an alternative to SB431542 with better *in vivo* exposure. GW788388 is orally active and has a good pharmacokinetic profile [13], [14], [30]. GW788388 administration reduced liver and renal fibrotic response in a model of chemically induced fibrosis in rats and in the db/db mouse model of spontaneous diabetic nephropathy [13], [14]. Treatment with GW788388 also showed efficacy for preventing the fibrotic response in a skin fibrosis model [33] and attenuated cardiac dysfunction following myocardial infarction [34]. These data prompted us to test this compound during the acute phase of experimental Chagas disease.

We found that oral administration of GW788388 at 3 dpi significantly reduced peripheral parasitemia and lowered parasite load in hearts of infected mice observed 15 dpi. This effect was achieved with lower administration doses (3 mg/kg) than the one we previously used for SB431542 (10 mg/kg) [12], and with a single oral administration. More importantly, oral administration of GW788388 also significantly improved mice survival (70% in GW788388-treated mice against 30% in non-treated infected mice at 30 dpi). This is probably due to the combined impairment of the second wave of *T. cruzi* parasitemia due the decrease of parasite burden and of the early inflammatory cytokines secretion balance. Infection with *T. cruzi* in the acute phase is followed by a strong mononuclear cell inflammation on target tissues such as heart and liver, which could cause tissue disruption, necrosis followed by fibrotic deposition and abnormalities in electrical impulse conduction. Our data showed less inflammation on both heart and liver tissues and, moreover, less mononuclear cells by inflammatory focus. An improved ECG profile was also observed after GW788388 administration, characterized mainly by the absence of sinus node dysfunctions and reduced sinus bradycardia. PR intervals larger than 40 ms suggested slower transmission of the electrical impulses and atrioventricular block (AVB), which is characteristic of acute *T. cruzi* infection [35]. We observed an improvement of the QT intervals following GW788388 administration, which represent the wave of ventricular recuperation and this could be related to the decrease of sudden death [36] and to the progression to a pathological chronic phase [35]. Heart failure and sudden death are the most common causes of death in patients with chronic cardiac Chagas disease [37] and altered ECG parameters correlates with increasing myocardial scar and decreasing myocardial function in these patients [38]. This results from disorganized gap junctions that could contribute to abnormal impulse conduction and arrhythmia that characterize severe cardiopathy in Chagas disease and heart fibrosis [10]. Gap junction Cx43 molecules are responsible for electrical impulse conduction in the heart [39] and are affected by TGFß [10], [40]. We observed that GW788388 treatment preserved a correct Cx43 plaque pattern in the heart and blocked the down-regulation of Cx43 expression commonly observed following *T. cruzi* infection. GW788388 treatment therefore favored a regular and correct electrical impulse transmission. TGFß is also a key factor in the generation of tissue fibrosis [41] and has been correlated to development of Chagas disease symptoms in cardiac chronic phase [8]. Our data showed that administration of GW788388 to *T. cruzi*-infected mice significantly prevented the increase of fibronectin and collagen type I, two important components involved in heart fibrosis. These data are consistent with previous studies showing that GW788388 reduced fibrosis markers in the kidney following chemically induced nephropathy [14], [42].

In the human acute phase of Chagas disease, symptoms are frequently mild and not noticed and it is therefore difficult to propose correct treatments with trypanocidal drugs. Therefore, in the present study, we also treated mice with GW788388 at the end of the acute phase, when there are scarce circulating parasites. Interestingly, we found that oral administration of GW788388 at 20 dpi completely protected mice from death (100% survival). Analysis of cardiac fibrosis by Masson's trichrome staining on heart cross-sections of *T. cruzi*-infected mice showed a strong increase of fibrosis from 15 dpi to 24 dpi (Fig. 5, Table 4). Interestingly, we found that mice treated with GW788388, in a single dose scheme at 20 dpi, reversed heart fibrosis observed four days later (24 dpi) as compared to untreated infected mice. The level of collagen type I was also restored in GW788388 treated mice versus untreated mice. Taken together these data demonstrated that blocking TGFß signaling could decrease an installed heart fibrosis. This important finding encourages further pre-clinical assays targeting fibrotic lesions that are always involved in the severity of the clinical picture observed in the chronic cardiac disease. The development of an efficient drug for Chagas disease is still a challenge and trypanocidal drugs such as nifurtimox and benznidazole are still the only drugs employed for specific Chagas disease treatment, although the observation of serious side effects. Treatment strategy approaching the reversion of fibrosis has been demonstrated here at the end of the acute phase of experimental Chagas disease. Still, further studies on a chronic experimental model are necessary previously to clinical assays. The inhibition of TGFß signaling pathway and its biological functions could then be considered as an alternative strategy for the treatment of the symptomatic cardiomyopathy found in the acute and chronic phases of Chagas disease, in synergy with current administered drugs, enabling lower dosages and avoiding toxic effects.

## Supporting Information

Figure S1 **Dose-dependent analysis of the effect of oral administration of GW788388 at 3 dpi on parasitemia and survival rates.** Male Swiss mice were injected ip. with 10^4^ bloodstream trypomastigotes. Then GW788388 (0.3–15 mg/kg) or vehicle (DMSO) was administered once by gavage at 3 dpi. (A) Parasitemia was measured by direct counting of parasites in blood. (B) Percent survival was monitored until 30 dpi.
(EPS)

Figure S2 **Effects of in vitro GW788388 administration to cardiomyocytes on** ***T. cruzi*** **invasion and replication.** Cardiomyocytes were infected with trypomastigotes of the Y strain in a parasite∶host cell proportion of 10∶1 and 24 h post- infection, cultures were treated or not with GW788388 (10 µM). Cells were fixed 48 h (A and B) and 96 h (C and D) post-infection and stained with Giemsa. Magnification: 400×. Quantification of the percentage of cardiomyocytes containing parasites (E) and the number of parasites per infected cell (F) were determined by counting 400 cells/slide on two distinct coverslips at 48 and 96 h post-infection.
(TIFF)

Methods S1 **GW 788388 dose-response effect in vivo.**
(DOCX)
